RETRACTED

# Anthropogenic Radio-Frequency Electromagnetic Fields Elicit Neuropathic Pain in an Amputation Model

**DOI:** 10.1371/journal.pone.0144268

**Published:** 2016-01-13

**Authors:** Bryan Black, Rafael Granja-Vazquez, Benjamin R. Johnston, Erick Jones, Mario Romero-Ortega

**Affiliations:** 1 Department of Bioengineering, University of Texas at Dallas, 800 W. Campbell Road, Richardson, TX, 75080, United States of America; 2 Alpert Medical School, Brown University, 222 Richmond St., Providence, RI, 02903, United States of America; 3 Department of Industrial, Manufacturing, and Systems Engineering, University of Texas at Arlington, 500 West 1st St., Arlington, TX, 76019, United States of America; University of Montreal, CANADA

## Abstract

Anecdotal and clinical reports have suggested that radio-frequency electromagnetic fields (RF EMFs) may serve as a trigger for neuropathic pain. However, these reports have been widely disregarded, as the epidemiological effects of electromagnetic fields have not been systematically proven, and are highly controversial. Here, we demonstrate that anthropogenic RF EMFs elicit post-neurotomy pain in a tibial neuroma transposition model. Behavioral assays indicate a persistent and significant pain response to RF EMFs when compared to SHAM surgery groups. Laser thermometry revealed a transient skin temperature increase during stimulation. Furthermore, immunofluorescence revealed an increased expression of temperature sensitive cation channels (TRPV4) in the neuroma bulb, suggesting that RF EMF-induced pain may be due to cytokine-mediated channel dysregulation and hypersensitization, leading to thermal allodynia. Additional behavioral assays were performed using an infrared heating lamp in place of the RF stimulus. While thermally-induced pain responses were observed, the response frequency and progression did not recapitulate the RF EMF effects. *In vitro* calcium imaging experiments demonstrated that our RF EMF stimulus is sufficient to directly contribute to the depolarization of dissociated sensory neurons. Furthermore, the perfusion of inflammatory cytokine TNF-α resulted in a significantly higher percentage of active sensory neurons during RF EMF stimulation. These results substantiate patient reports of RF EMF-pain, in the case of peripheral nerve injury, while confirming the public and scientific consensus that anthropogenic RF EMFs engender no adverse sensory effects in the general population.

## Introduction

Anthropogenic electromagnetic fields (EMFs) have become a ubiquitous presence in modern life. A broad spectral band of EMF frequencies (50 Hz–5 GHz) are now passing around us and through us, and are generated by sources ranging from electricity transport to mobile communication devices. While we have all undoubtedly benefited from the wide-ranging applications of commercial electronics, there is a growing social and scientific concern that persistent exposure to radio- and microwave-frequency (RF/MWF) EMFs may engender unforeseen adverse health effects in vulnerable subsets of our population.

RETRACTED

Over the past thirty years, there have been numerous reports published on the epidemiological, animal, and cellular-level effects of RF EMF exposure [1–3], with the majority of these studies being conducted *in vitro* and focused on evaluating the potential relationship between cell phone usage and the incidence of certain types of cancer [4–6]. Many conclusions drawn from this field of study remain highly controversial [7,8], but sufficient evidence regarding EMF-tissue interactions has resulted in the adoption of national and international standards for health and occupational EMF exposure. More recently, there have also been anecdotal, case, and clinical reports that magnetic and electromagnetic fields of various frequencies may serve as a trigger for neuropathic and post-amputation pain [9–11].

Whether anthropogenic RF EMFs are capable of triggering post-neurotomy pain is a question of enormous clinical importance, as there are currently 1.7 million amputees living in the United States alone. Aside from the loss of function, approximately 20–30% of this population endures chronic, debilitating pain associated with the formation of benign peripheral nerve tumors in their residual limbs, called amputation neuromas [12]. This type of neuroma is the result of regenerating and sprouting axons, which grow into surrounding connective tissues following nerve transection. The resulting neuroma bulb, which is comprised primarily of unmyelinated and thinly myelinated (C and Aδ) nerve fibers, is well-known to respond to chemical, mechanical, and thermal stimuli with hypersensitivity [12–14]. However, to date, there has been no independent, reproducible confirmation that anthropogenic RF EMFs elicit post-neurotomy pain in either humans or animal models.

Here, we evaluate the claim that anthropogenic-strength RF EMFs are capable of eliciting post-neurotomy pain by adopting a modification of the tibial neuroma transposition (TNT) model for behavioral assessment of post-neurotomy pain in rats. Adult Wistar rats were randomly assigned to either receive the TNT or SHAM surgical procedure. Researchers blinded to the surgical groups then scored pain responses on a graded scale as animals were exposed to a circularly polarized RF antenna (915 MHz at 756 ± 8.5 mW/mm^2^). Measurements of skin temperature during RF EMF exposure revealed a transient increase of 2.1 ± 0.7°C during stimulation. We hypothesized that RF EMF-induced pain responses may be attributable to thermal allodynia, which results from the local secretion of inflammatory cytokines, such as tumor necrosis factor alpha (TNF-α) and interleukin 1-beta (IL-1β). Both TNF-α and IL-1β have been shown to contribute to allodynia [15,16] and thermal hyperalgesia [17] through the dysregulation of temperature-sensitive channel expression [18–20], such as members of the transient receptor potential (TRP) family. Histological staining for TRPV4, a non-selective cation channel which is highly implicated in thermal sensation and various neuropathic pain states [21–23], was carried out in neuroma and uninjured tibial nerve sections. In parallel, calcium imaging experiments were conducted on dissociated dorsal root ganglion (DRG) neurons in the presence and absence of TNF-α in order to determine whether the RF EMF stimulus was sufficient to directly depolarize sensory neurons. Our findings confirm that RF EMFs are capable of eliciting post-neurotomy pain in an animal model.

RETRACTED

## Results

### RF EMFs elicit post-neurotomy pain

Twenty female adult Wistar rats were divided into two groups. Sixteen animals underwent the TNT procedure, while the remaining 4 animals received a SHAM surgery, as described in ‘Methods’. The TNT surgery resulted in neuroma bulb formation in all animals as exemplified in Fig 1B. Following TNT and SHAM surgeries, animals were coded and individually exposed to a circularly polarized RF EMF antenna (915 MHz at 756 ± 8.5 mW/m^2^) for 10 minutes, once per week for 8 weeks. The RF EMF stimulus was attenuated to deliver an average power density equal to that measured at 39 m from a local cell phone tower (763 mW/m^2^ at 39 m; S1 Fig), which we selected as an example of the maximum anthropogenic EMF power density a person might encounter outside of select occupational settings.

**Fig 1:** The modified tibial neuroma transposition (TNT) surgery and RF EMF behavioral response assays. (A) Depiction of the TNT surgery. The three distal branches of the sciatic nerve (tibial: blue, sural: red, and common peroneal: yellow) were teased from the surrounding connective tissue and from each other. The tibial branch was then transected (black X) and transposed from its original (dashed blue line) to its final orientation (solid blue line), and sutured to the fascia adjacent to the hip bone (black dashed line). TNT surgery resulted in neuroma formation. (B) 8 week old neuroma bulb. Separation between black lines equals 1 mm. (C) Representative image of a Wistar rat during (C) baseline and (D) stimulus period (10 minutes at 756 ± 8.5 mW/mm^2^) of the RF EMF (915 MHz) behavioral assay. Animal presents a left hind limb withdrawal. This action represents a response score of 1. (E) Timeline for surgical procedures (S1 and S2) and behavioral response assays.

RETRACTED

The summed response score for each animal is plotted as a function of time in Fig 2A and 2B. Beginning on postoperative week 1, 47% of animals from the TNT group exhibited at least one pain response during RF EMF stimulation. By postoperative week 4, this percentage increased to 88%, which is consistent with expected neuroma growth and sensitization. In sharp contrast, only one animal from the SHAM group exhibited a single behavioral response during RF EMF stimulation, observed at week 1. No additional pain responses in the SHAM group were observed. The mean response score for the TNT group differed significantly from the SHAM group beginning on postoperative week 3 (p = 0.049) and persisting on week 4 (p = 0.006). These results demonstrate for the first time that anthropogenic-strength RF EMFs are sufficient to trigger post-neurotomy pain in a behaving animal model.

**Fig 2:** Radio-frequency electromagnetic field (RF EMF) stimulation elicits post-neurotomy pain. (A) Hollow circles indicate the summed response score for each animal for both TNT (red) and SHAM (grey) groups. Only one behavioral pain response was observed in the SHAM group over all 10 experimental trials. Statistically significant mean response scores (solid black line) were observed between TNT and SHAM groups beginning in week 2 and continuing through week 8. Lidocaine was found to be a successful moderator of RF EMF-induced neuroma pain. Dashed black lines indicate population median. (B) Following bulb resection surgery, significant RF EMF-induced neuroma pain persisted from week 5 until week 28. For statistical comparisons, a two-tailed Mann-Whitney test was used (* p<0.05, ** p<0.01). (C) RF EMF exposure induces mean skin temperature increase. A mean skin temperature increase of 2.2°C was observed following 10 minutes of RF EMF exposure. (D) Recovery/Stimulus behavioral response ratios for all time points.

To confirm that pain responses were nerve-mediated, RF EMF assays were carried out one day following week 4 assays while nerve conduction was blocked by a subdermal injection of lidocaine (100 μl, 1 g/ml), administered at the neuroma site. The mean response score of the TNT group was significantly reduced following lidocaine injection when compared to week 4 response scores (p = 1.16 x 10^−4^). These results demonstrate that RF EMF-induced pain response is the result of depolarizing nerve activity.

### RF EMF-induced pain is chronic and persists following neuroma bulb resection

One day following Lidocaine trials, animals from the TNT group were randomly divided into two additional groups: TNT-SHAM (TNT-S, N = 8) and TNT-Bulb Resection (TNT-BR, N = 8). TNT-BR animals underwent surgery to dissect and remove the neuroma bulb. TNT-S animals and SHAM-S animals received identical pre- and post- operative treatment, but did not have their neuroma bulbs removed or their tibial nerves transected, respectively. Pain response assays resumed for weeks 5–8 from the date of initial TNT surgery and were repeated on one additional, chronic time point (week 28).

RETRACTED

Surprisingly, RF EMF-induced pain responses persisted in weeks 5–8 for animals in both the TNT-S and TNT-BR groups, while no pain responses were observed in the SHAM-S group in weeks 5–8 or on week 28 (Fig 2B). The mean response scores for the TNT-S and TNT-BR groups both differed significantly from the SHAM-S group consistently from week 5 onward. While there was no significant difference between the mean response scores of the TNT-S and TNT-BR groups in weeks 5–8, the two groups differed significantly in week 28. At this point, the TNT-S group showed pain responses similar to those observed in the first four weeks of the study, whereas the TNT-BR group showed significantly higher pain responses (p = 0.005). These results suggest that neuroma bulb resection may not be an effective intervention for RF EMF-induced post-neurotomy pain in either the short- or long-term. In fact, it may exacerbate post-neurotomy pain by introducing a second injury to the nerve.

### RF EMFs induce an increase in skin temperature

Skin temperature measurements were acquired by laser-thermometer (TW2, ThermoWorks, USA) from 10 randomly selected animals during 10 minute baseline (antenna off), stimulus (antenna on), and recovery (antenna off) intervals. During the stimulus interval, we measured a mean transient skin temperature increase of 2.1 ± 0.7°C, which returned to near-baseline levels (31.5 ± 2.2°C) during the recovery interval (Fig 2C). Therefore, all animals were observed for an additional 10 minutes following stimulus in order to account for residual response scores during tissue cooling. Fig 2D shows the ratio of Recovery/Stimulus response scores as a function of time. This ratio continuously increased from 0.43 in week 1 to 0.92 in week 4. Following the second surgery, the Recovery/Stimulus ratio is again comparable to week 1 (0.48) and increases over time until week 8 (0.65). Importantly, this data serves as a secondary confirmation that pain responses are due to RF EMF stimulation, as the summed stimulus-interval pain score is consistently and considerably higher than that of the recovery interval. Furthermore, this data suggests that the second surgical procedure partially disrupts the mechanism responsible for increasing residual pain response through the first 4 weeks.

RETRACTED

### Thermal stimulus elicits post-neurotomy pain, but does not completely recapitulate the RF EMF effects

In order to compare RF EMF-exposure to direct thermal stimulation (a known trigger for post-neurotomy pain), animals were individually exposed to a 125 W infrared heating source for 5 minutes, once per week for 8 weeks. Exposure to the infrared source resulted in a transient mean skin temperature increase of 4.8 ± 0.4°C above baseline. From postoperative week 1 to week 4, the percentage of TNT animals which exhibited at least one behavioral response during thermal stimulation increased from 19% to 50%. Pain responses persisted over all 4 weeks and the mean response score increased each consecutive week through week 4 (Fig 3A), consistent with neuroma growth. No animals from the SHAM group exhibited even a single behavioral response to the thermal stimulus throughout the duration of the study. Lidocaine injection was found to be somewhat effective in reducing pain response, though the difference was not statistically significant. These findings are in agreement with previous reports that temperatures below what would typically be perceived as noxious heat stimuli (> 47°C) are capable of triggering neuroma pain. It is important to note, however, that direct thermal stimulation was less effective at eliciting post-neurotomy pain when compared to RF EMF (i.e. 50% versus 80% response by week 4), even at a higher temperature increase (4.8°C versus 2.1°C). This suggests that, while there may be a component of RF-induced neuroma pain attributable to temperature, additional mechanisms may be involved.

**Fig 3:** Thermal stimulus elicits post-neurotomy pain. (A) Hollow circles indicate the summed behavioral response score for each animal for both TNT (red) and SHAM (grey) groups. Statistically significant mean pain response scores (solid black line) were observed between TNT and SHAM groups in week 4 and in weeks 6–8, following bulb resection (B). Lidocaine was found to be a successful moderator of heat-induced neuroma pain. Dashed black lines indicate population median. (B) Following bulb resection surgery, significant heat-induced neuroma pain persisted from week 6 until week 28. No statistically significant difference was found between animals receiving bulb resections vs TNT-SHAM animals. For statistical comparisons between groups, a two-tailed Mann-Whitney test was used (* p<0.05, ** p<0.01). (C) Thermal stimulus exposure induces a significant mean skin temperature increase. A mean skin temperature increase of approximately 5°C was observed following 5 minutes of heat-lamp exposure. (D) Recovery-to-Stimulus behavioral response ratios for all time points.

RETRACTED

### Temperature-induced pain is persistent following neuroma bulb resection

Temperature-evoked pain persisted in the TNT-S and TNT-BR groups throughout the duration of the study, while no pain responses were observed in the SHAM-S group (Fig 3B). The mean response scores for the TNT-S and TNT-BR groups differed significantly from the SHAM-S group beginning on week 6 and persisting through week 8 (p < 0.05), yet there was no significant difference between TNT-S and TNT-BR groups in week 5–8 or week 28. These results indicate that bulb resection exacerbates post-neurotomy pain over the short term, with pain scores returning to pre-resection values between weeks 8 and 28.

### Thermal stimulation induces residual pain

To account for the potential effects due to delays in skin temperature cooling (Fig 3C), pain responses were scored for an additional 5 minutes, referred to here as the ‘Recovery’ interval. As expected, direct thermal stimulus resulted in residual pain responses during the recovery interval. In general, the Recovery/ Stimulus ratio for thermal stimulation was higher than for RF EMF stimulation at each time point, with this value exceeding 1 on weeks 3 and 5 (Fig 3D). This is likely correlative to delayed cooling caused by greater temperature increase. Additionally, the time dependence trend of the thermal Recovery/Stimulus ratio does not follow that of the RF EMF, implying that a different functional mechanism is responsible for residual responses in the case of the two stimuli.

### Neuroma formation results in increased expression of TRPV4 channels

Our previous results suggested that RF EMF-induced pain is mediated by thermal allodynia. Allodynia following nerve transection results from the local secretion of inflammatory cytokines, such as tumor necrosis factor alpha (TNF-α) and interleukin 1-beta (IL-1β). Both TNF-α and IL-1β have been shown to contribute to allodynia [15,16] and thermal hyperalgesia [17], specifically through the dysregulation of temperature-sensitive channel expression [18–20], and the heat-potentiation of sensory afferents [20,24]. Several families of temperature-sensitive ion channels are subject to such dysregulation, including members of the TRP family. Since the temperature increase associated with RF EMF stimulus is not tantamount to a noxious heat stimulus, we hypothesized that TRPV4 channels may be involved, as these channels are expressed in sensory nerve afferents and dorsal root ganglia, are activated by temperature ramps within the physiological range (< 40°C), and are implicated in neuropathic pain [21,25].

RETRACTED

We confirmed by immunolabeling of 8 week old neuromas a four-fold increase in the expression of TRPV4 channels in the neurom bulb (1.7 X 10^5^ puncta/mm^2^; p < 2.1 X10^-9^) versus the contralateral healthy tibial nerve (0.4 X 10^5^ puncta/mm^2^; Fig 4G). As expected, DAPI staining showed a significant recruitment of non-neuronal cells to the neuroma bulb compared to the healthy tibial nerve (Fig 4G). This data suggests that RF EMF-induced postampuation pain may be mediated by thermal activation of TRPV4 channels.

**Fig 4:** Increased expression of TRPV4 channels and recruitment of non-neuronal cells in 8-week-old amputation neuroma. Representative confocal images (60x with 2x scan zoom) of DAPI-stained cell nuclei ((A, D), blue) and TRPV4 channels ((B, E), gold) in uninjured tibial nerve tissue and within the neuroma bulb, respectively. Scale bar represents 15 μm. (G) Mean density of nuclei and TRPV4 channels (puncta) in uninjured tibial and neuroma tissues (n = 12). Density comparisons were made by 2 sample t-test (** p<0.01).

### RF EMF evokes higher-threshold calcium spikes in dissociated DRG neurons

The cellular mechanism by which tissue heating, particularly in combination with nerve injury, elicits pain may involve a number of different cells including macrophages, Schwann cells, fibroblasts, as well as sensory axons. In order to determine whether RF EMF stimulus is sufficient to modulate the spontaneous activity of primary sensory neurons, we performed calcium imaging experiments on dissociated DRG neurons. The cells were incubated with Fluo-3 and imaged at 1 Hz (20x, 488 nm excitation) in an environmentally controlled (37°C, 5% CO_2_) stage-top incubator, 7 days following culture. The evaluation intervals followed those used in the behavioral assays (2 minute baseline, 10 minute stimulus, and 10 minutes recovery). As a negative control, calcium imaging experiments were also conducted with no RF EMF applied (Fig 5).

**Fig 5:** Effects of RF EMF on the spontaneous spiking activity of dissociated DRG sensory neurons in the absence and presence of inflammatory cytokine, TNF-α. (A) Representative confocal image of dissociated DRG neurons following 15 min incubation with 5 μM Fluo-3 AM (Scale bar = 15 μm). (B) Unsmoothed ΔF/F for a single cell. Spikes correlate to an increase in intracellular calcium concentration. (C) Spikes per active cell calculated at 0.35 for RF EMF ‘OFF’ (n = 163) or ‘ON’ (n = 232). Spikes persisted after removal of the RF stimulus, which was consistent with observations from behavioral assays. (D) A larger percentage of DRG neurons were active when RF EMF stimulus was applied to cultures perfused with inflammatory cytokine TNF-α (10 ng/ml).

RETRACTED

Fig 5A is a representative image of dissociated DRG neurons following incubation with Fluo-3. ΔF/F plots (Fig 5B) revealed that spontaneous spikes in intracellular calcium concentration were common in cases of No RF as well as when RF was applied. A significantly higher spiking rate was observed when RF EMF stimulus was applied (spike threshold = 0.35, Fig 5C). This result suggests that RF EMF stimulation is sufficient to directly elicit higher threshold activity in dissociated DRG neurons without functional sensitization.

### RF EMF-induced depolarization is exacerbated by TNF-α

In order to better simulate the conditions of inflammatory injury, calcium imaging experiments were also conducted in the acute and chronic presence of inflammatory cytokine, TNF-α. In acute experiments, TNF-α was perfused into the DRG culture over 1 minute to reach a final concentration of 10 ng/ml. This concentration has been shown to cause increased sensitivity in both acute and chronic applications. A 25% percentage increase in the number of spiking cells in response to RF EMF + TNF-α (Fig 5D) at minute 4 was observed. The increased values induced by TNF-α were statistically different as indicated by a Paired Wilcoxon Signed Rank Test (p = 0.03). In chronic experiments, DRG neurons cultured with TNF-α for 50 hours showed an increased average spiking rate and amplitude compared to acute or control experiments. However, no significant difference in spiking rate, spiking amplitude, or active cell percentage was observed between the RF Applied and No RF groups (data not shown). These results suggest that RF EMF in combination with acute TNF-α results in a greater number of active sensory neurons, but that chronic exposure to this cytokine alone is not sufficient to cause RF EMF hypersensitivity.

It has been shown that calcium activity among glial cells can modulate the activity threshold of surrounding sensory neurons. Therefore, modulated resting potentials for non-neuronal cells may affect potentiation of sensory neurons. S2A–S2H Fig shows two sets of non-neuronal DRG cells present in cultures during chronic TNF-α calcium imaging experiments. The intracellular calcium concentration of these cells was found to gradually shift throughout the duration of RF EMF exposure. Cells shown in S2A–S2D Fig exhibited an approximate 150% increase in fluorescence intensity, while cells shown in S2E–S2H Fig exhibit a nearly 100% decrease in fluorescence intensity. Such dramatic and sustained shifts in intracellular calcium concentration baselines among non-neuronal cells during and following RF EMF stimulation may influence the activity of adjacent sensory neurons *in vivo*.

RETRACTED

## Discussion

The World Health Organization (WHO) and the International Commission on Non-Ionizing Radiation Protection (ICNIRP) have adopted occupational and environmental EMF exposure thresholds based on a tissue or organ system’s specific energy absorption rate (SAR) [26]. Therefore, current safety standards are closely related to a tissue’s temperature rise due to direct EMF absorption. However, these standards and guidelines largely disregard potential effects suffered by those subject to injured or malfunctioning tissues. To date, clinical or case reports of EMF-induced post-neurotomy or neuropathic pain have been widely dismissed. This is likely due to the fact that numerous provocation studies have been conducted addressing the anecdotal self-reporting of electro-magnetic hypersensitivity among the general population. These studies have provided no evidence that those with reported EMF hypersensitivity are able to detect the presence of EMFs or that they suffer any physiological stress during EMF provocation trials [27,28].

For the first time, in a blinded animal study, we have confirmed anecdotal reports that anthropogenic RF EMFs are capable of triggering post-neurotomy pain. Furthermore, we have confirmed that RF EMF-induced pain signaling is, in part, nerve mediated, as pain was successfully interrupted by local lidocaine anesthesia. However, the fact that RF EMF pain was induced as early as postoperative week 1 suggests that pain responses are not completely dependent on the formation of a ‘matured’ neuroma bulb, since painful neuromas typically require several weeks, or even months, to form and become symptomatic. For the same reason, it is also unlikely that pain responses are due to ephaptic cross talk between regenerated unmyelinated nerve fibers at the site of the neuroma bulb. These results do not, however, rule out the contribution of neuroma formation in the progression of RF EMF pain. On the contrary, it clarifies the fact that neuropathy results in a massive disruption of the perineurium, exposing nerve fibers to inflammatory cytokines and exacerbating pain response in the acute inflammatory phase following amputation. This initial inflammatory response decreases with time as the blood-nerve barrier is re-established. Her we show that developed neuromas are comprised mostly of thinly and unmyelinated axons, which expressed heightened levels of TRPV4 channels. These non-specific cation channels are dysregulated and hypersensitized following exposure to inflammatory cytokines such as TNF-α and IL-1β, and can therefore mediate thermal allodynia due to even mild temperature increases. This type of alteration in channel expression and function is not exclusive to nerve transection injuries. Therefore, this study suggests that the criteria for RF EMF sensitization may be satisfied by other types of acute and/or inflammatory nerve injury and a more general category of neuropathic pain states.

RETRACTED

Our findings that a 915 Hz RF EMF stimulus elicits pain in acute nerve injuries, as well as in developing neuromas, suggests that this approach may be an effective tool for the diagnosis of developing neuropathic hypersensitivity and serve as an early endorsement for post-neurotomy intervention strategies. To fully determine the use of this approach as a diagnostic tool, future studies should compare this type of RF EMF to other available technologies such as transcranial magnetic stimulation (TMS), which has been shown to be an effective tool for diagnosing ‘active’ stump neuroma following amputation surgery [29].

In vitro experiments demonstrated that DRG sensory neurons are directly susceptive to a significant increase in the frequency of high-threshold calcium transients during RF EMF stimulus. Importantly, this response was exacerbated by the presence of inflammatory cytokine TNF-α, as a higher percentage of DRG neurons were active during RF EMF stimulus. This suggests that several, decentralized mechanisms may be activated in concert by RF EMF stimulus; both thermal and athermal. Recently, several athermal effects of RF EMF exposure have been reported, including the upregulation of heat shock proteins [30], decreased cell proliferation [31], DNA damage [32], and proteome alterations [33]. The conclusiveness of these athermal findings, however, has suffered from a lack of independent reproducibility, most probably associated with the lack of consistent dosimetry in what is still a burgeoning field of study [34,35]. This is especially important since the few existing systematic parametric studies suggesting therapeutic or deleterious effects of EMFs report that these effects occur within both amplitude and frequency ‘windows’ [6,36]. One such study demonstrated that room temperature application of 915 MHz EMF resulted in significant condensation of chromatin, closely mimicking the effects of heat shock (at 41°C) [36].

## Conclusion

Our animal study supports anecdotal reports indicating that RF EMFs serve as a trigger for post-neurotomy pain. Further, it suggests that those who have suffered a nerve injury or other types of peripheral nerve pathology may be prone to RF EMF-induced pain. The fact that uninjured animals showed no response to RF EMF in this study is also in agreement with most scientific reports and the overwhelming view that, under normal circumstances, anthropogenic EMFs in the reported range causes no pain. Thus, this study offers a possible explanation for contradicting accounts on evoked pain by RF EMF and highlights nerve pathology as the crucial contributing factor to RF EMF-induced symptoms. These findings may prove valuable in developing a patient’s pain management protocol and inform future studies of EMF-pain phenotyping.

RETRACTED

## Materials and Methods

### Animal model and TNT surgery

In order to simulate amputation in a behaving animal model, we have adopted a modification of the tibial-neuroma transposition surgery described in Dorsi, et al [37]. Our reasons for modifying the surgical procedure put forth by Dorsi, et al were two fold. (1) We believed that approaching the sciatic nerve through the separation in the vastus lateralis and biceps femoris made for a less aggressive procedure, since it did not ultimately require tunneling through tissues to access the tibial branch translocation point. (2) Thermal and RF EMF behavioral response assays were predicated on field absorption. It was, therefore, desirable for the transected tibial translocation position to be more ‘accessible’ to the stimuli. From 20 Wistar rats, 16 were randomly selected to receive the tibial-neuroma transposition (TNT) surgery, and the remaining animals (N = 4) received SHAM surgeries, as described in the following section.

Briefly, animals were anesthetized with 1.5% isoflurane and the left thigh was shaved and sterilized with 70% ethanol and povidone-iodine. A lateral incision was made in the left hind limb, starting approximately two centimeters caudal to the hip bone and in a plane parallel to the femur. The vastus lateralis and biceps femoris muscles were separated, exposing the sciatic nerve, and approximately one centimeter of the tibial branch was isolated. The tibial branch was transected at the level of the popliteal artery and transposed atop the quadriceps muscle, adjacent to the hip bone, and fixed with a 9–0 nylon suture. We then affronted the biceps femoris with chromic gut thread and the skin was closed with stainless steel staples.

The remaining animals (N = 4) received a SHAM surgical procedure, wherein the tibial nerve was exposed, but not transected. All animals received identical pre- and post-operative care, which included postoperative application of triple-antibiotic ointment, an injection of sustained-release buprenorphine (1 mg/kg SC, QTD), and daily injections of prophylactic antibiotic (Cefazolin, 1 mg/kg IM) for one week. Animals were housed, one animal per cage, in a climate controlled room (60% humidity) under a 10:14 hr light/dark cycle, with free access to suitable food and water. The health and well-being of all animals was monitored daily by research staff and once per week by a veterinarian. Following the completion of behavioral assays, animals were sedated by 1.5% isoflurane and euthanized by injection of sodium pentobarbital (120 mg/kg). All handling and housing measures, surgical procedures, and behavioral assays were approved by the University of Texas at Arlington and the University of Texas at Dallas Institutional Animal Care and Use Committee.

RETRACTED

### Behavioral response scoring

Behavioral response assays began one week following surgical procedures, and were conducted on the same day of each week for 8 consecutive weeks plus one chronic time point (week 28). All animals were number-coded and researchers were blinded. Behavior was graded on a range from 0 to 2, as previously described [37]. Briefly, a grade of 0 indicates no response. A grade of 1 was assigned for a withdrawal of the left hind limb. A grade of 2 was assigned for prolonged left hind limb extension (more than 1 second), shaking or licking of the left hind limb, or a vocalization (S1 Video). The reported ‘response score’ represents the sum of the individual graded responses observed during RF EMF or thermal stimulation.

### RF EMF stimulation

Animals were individually placed into a clear acrylic box with a RF antenna (915 MHz, Andrew RFID-900-SC) fixed approximately 10 in. (25.4 cm) above, with ample clearance for air exchange. The antenna was attenuated to deliver a time-averaged maximum power density of 756 ± 8.5 mW/m^2^, as measured by a 3-axis RF field-strength meter (TM-196, Tenmars, Taiwan). This power density was selected based on maximum field-strength measurements conducted near an active cell-phone tower in our area (S1 Fig). In conjunction, we measured the external electric field to be 21.5 ± 0.1 V/m, which corresponds to a SAR of 0.36 W/kg at the skin surface. While this does not consider the contribution of induced electric fields inside the tissue, this SAR is approximately 4 times less than currently advised maximum permissible exposure (1.6 W/kg, spatial peak) for general populations [38]. RF EMF behavioral response assays consisted of three experimental intervals: 2 minutes of baseline (antenna off), 10 minutes of RF stimulation (antenna on), and 10 minutes of recovery (antenna off). RF EMF power density during ‘antenna off’ intervals was measured to be approximately 350 μW/m^2^. The total ‘behavioral response score’ was taken as the sum of each behavioral response over the RF EMF stimulation period.

RETRACTED

In order to determine whether a transient temperature rise might occur during RF EMF stimulation, laser-thermometer skin temperature measurements were taken from 10 randomly selected animals prior to undergoing surgical procedures. During the ‘antenna on’ interval, a mean skin temperature increase of 2.1 ± 0.7°C was observed, which returned to near-baseline levels during the recovery interval (Fig 2C). Additionally, core body temperature measurements (N = 4) indicated no significant temperature difference (-0.3 ± 0.1°C) during RF EMF exposure, illustrating that RF EMF-induced temperature increase is both transient and localized.

### Thermal stimulation

In order to characterize the pain response evoked by direct thermal stimulation, a skin temperature difference of approximately 5°C was induced by exposure to an infrared heating lamp. Animals were individually placed into a clear acrylic box with a 125 W infrared lamp (Philips, Korea) positioned 12 inches (30.5 cm) above the animal. Pain responses were evaluated during three experimental intervals: 2 minutes of baseline (heat lamp off), 5 minutes of thermal stimulation (heat lamp on), and 5 minutes of recovery (heat lamp off). The thermal stimulation duration was selected in order to achieve a mean skin temperature rese of approximately 5°C from baseline, and was determined by laser-thermometer measurements conducted on 10 randomly selected animals prior to TNT surgeries.

### Lidocaine block of nerve conduction

Lidocaine control assays were conducted one day following ‘Week 4’ behavioral response assays. Each animal was lightly anesthetized using 2% isofluorane and received a subdermal injection of 100 μL 2% Lidocaine at the neuroma site. Approximately 10 minutes after recovering from anesthesia, each animal was subjected to behavioral response assays, as described above.

### Dorsal root ganglion culture and calcium imaging

All *in vitro* calcium imaging experiments were performed on dissociated embryonic (E 16–18) dorsal root ganglion (DRG) neurons. Whole embryonic mouse DRGs were purchased from BrainBits, Inc. (BrainBits, USA) and were enzymatically dissociated by incubation with 1 mg/ml collagenase (Invitrogen, USA) at 37°C for 60 min. DRGs were then transferred to 0.125% Trypsin (Sigma Aldrich, USA) and incubated at 37°C for 15 min. Trypsinization was quenched by adding 10% fetal bovine serum in Hank’s Buffered Salt Solution (Sigma Aldrich, USA) and further mechanical dissociation was carried out by 30x gentle trituration using a sterile glass fire-polished Pasteur pipette. The dissociated tissue was collected by centrifugation at 200 g for 3 min. DRG neurons were then re-suspended in NbActiv4 (BrainBits, USA) plus 25 ng/ml nerve growth factor (NGF, Sigma Aldrich, USA) and transferred onto glass-bottomed 35 mm culture dishes (In Vitro Scientific, USA), which had previously been coated with 0.1 mg/ml Poly-D-lysine (Sigma Aldrich, USA). Dissociated DRG cultures received 50% medium exchange (NbActiv4 plus 25 ng/ml NGF) every 3 days, and were housed continuously at 37°C and 5% CO2 prior to imaging. For visualization of intracellular calcium concentrations, dissociated DRGs were incubated for 15 minutes at 37°C with 5 μM Fluo-3 AM (an established cell-permeant Ca^2+^ indicator) in 250 μL NbActiv4. Cells were washed once with NbActiv4 and the medium was replaced before imaging. All fluorescence calcium imaging experiments were performed on a Nikon A1R confocal microscope system (Nikon, Inc.). Throughout the experiments, cells were housed in an environmentally controlled stage-top incubator (Tokai HIT) at 37°C and with 5% CO_2_. The RF antenna was fixed approximately 6 inches above the stage-top incubator. RF EMF dosage (756 ± 8.5 mW/m^2^ at 915 MHz) and exposure schedule (2 minute baseline, 10 minute RF exposure, and 10 minute recovery) were identical to those used in behavioral response assays.

RETRACTED

Within each culture dish, a field of view was selected which included 20–60 individually distinguishable fluorescent DRG neurons. Fluo-3 fluorescence was excited by a 488 nm laser diode, and the cells were imaged at 1 Hz across all experimental intervals. Individual sensory neuron cell bodies were outlined and defined as regions of interest (ROIs) within Nikon’s ND Elements software (Nikon, USA). Mean pixel intensity values were measured for all time-series data sets and ΔF/F values were calculated by establishing and subtracting a time-dependent fluorescence baseline for each cell, as previously described [39]. Peak detection was carried out in Matlab software, with the calcium spike threshold criteria set to ΔF/F ≥ 0.15 (unless otherwise indicated). Quantitative analysis of calcium spike frequency was carried out in novel Python script and statistical analysis was carried out in OriginPro 9.0 software (Origin Software, USA).

### Calcium imaging in the presence of TNF-α

In order to evaluate the potential synergistic effects of inflammatory cytokines and RF EMFs on dissociated DRG neurons, calcium imaging experiments were conducted in the acute and incubated presence of tumor necrosis factor-alpha (TNF-α, N = 95). Acute synergistic calcium imaging experiments consisted of four experimental intervals: 2 minutes of baseline (antenna off), 1 minute of cytokine perfusion (to a final concentration of 10 ng/ml), 10 minutes of RF stimulation (antenna on), and 10 minutes of recovery (antenna off). Incubated synergistic calcium imaging experiments were conducted following 50 hr incubation of DRG neurons in 10 ng/ml TNF-α and consisted of three experimental intervals: 2 minutes of baseline (antenna off), 10 minutes of RF stimulation (antenna on), and 10 minutes of recovery (antenna off).

RETRACTED

## Supporting Information

S1 Fig Measured EMF power density (mW/mm^2^) as a function of separation between the field meter and a local cell-phone transmission base tower. The yellow, highlighted circle indicates the highest measurement recorded within 50 meters of the tower’s base (763 mW/mm^2^). The dashed line indicates our chosen power density (750 mW/mm^2^), selected to mimic the maximum base station exposure.
(TIF)

S2 Fig On/off calcium levels observed in response to RF EMF stimulus. (A-D) Non-neuronal cells exhibiting sustained intracellular calcium influx. Image (A) shows the baseline fluorescence intensity, 2 minutes prior to initiating the RF EMF stimulus. Images (C-D) illustrate the sustained increase, which persisted after RF EMF stimulus was turned off (10 min). (E-H) Possible microglia exhibiting sustained calcium efflux following perfusion of 10 ng/ml TNF-α (at 0 min). Significantly reduced intracellular calcium concentration was sustained throughout experimental interval (22 min).
(TIF)

S1 Video Representative video of behavioral response in the presence of RF EMF stimulus. A grade of ‘1’ was given to withdrawal of the operated hind limb. A grade of ‘2’ was assigned for prolonged left hind limb extension (more than 1 second), shaking or licking of the left hind limb, or a vocalization. No behavioral response received a grade of ‘0’. Reported behavioral response scores reflect the sum of all response grades within the stimulus period.
(WMV)
